# Analysis of Risk Factors for Rheumatoid Arthritis in Yunnan: A Small-Scale Case-Control Study

This article has been retracted.

**DOI:** 10.1155/2022/3948448

**Published:** 2022-06-23

**Authors:** Wenrun Li, Yi Sun

**Affiliations:** Department of Medical Laboratory, The First People's Hospital of Yunnan Province, The Affiliated Hospital of Kunming University of Science and Technology, Kunming, Yunnan, China

## Abstract

**Objective:**

To study the risk factors of rheumatoid arthritis (RA) in Yunnan and provide reference for its clinical prevention and treatment.

**Methods:**

From January 2014 to February 2022, a total of 249 RA patients who were admitted to the First People's Hospital of Yunnan Province were selected and 149 healthy people were selected as the controls. The medical records, clinical data of blood test results of anticyclic citrullinated polypeptide (anti-CCP) antibody, antikeratin antibody (AKA), and antiperinuclear factor (APF) were collected. Logistic regression and receiver operating curve (ROC) were used to analyze the correlation between blood anti-CCP antibody, AKA, and APF and the occurrence of RA.

**Results:**

Univariate analysis showed that the age, proportion of hypertension, and diabetes patients in RA patients were significantly different from those in the control group (*p* < 0.05), but there was no statistical difference in sex (*p* > 0.05). The area under the curve (AUC) of the serum anti-CCP antibody level in the diagnosis of RA was 0.76 (95% CI: 0.72–0.81, *p* < 0.01), the sensitivity was 85.23%, the specificity was 61.45%, and the cutoff value was 18.07AU/mL. The positive rates of AKA (33.73%) and APF (43.37%) in the RA patients were significantly higher than those in the controls (4.03% and 6.04%), and the differences were statistically significant (*p* < 0.001). After adjusting for age, sex, hypertension, and diabetes, logistic regression analysis showed that anti-CCP positivity, AKA positive, and APF positive were all independent risk factors for RA (OR = 20.24, 95% CI: 9.36–43.77, *p* < 0.01; OR = 4.33, 95% CI: 1.62–11.60, *p* < 0.01; OR = 5.28, 95% CI: 2.33–11.99, *p* < 0.01).

**Conclusion:**

Anti-CCP positive, AKA positive, and APF positive are independent risk factors for the occurrence of RA. Serum anti-CCP level has high sensitivity but low specificity in the diagnosis of RA.

## 1. Introduction

Rheumatoid arthritis (RA) is one of the most common autoimmune diseases characterized by autoantibody production, synovial inflammation, cartilage destruction, and bone erosion [1]. Due to the complexity of the pathogenesis of RA, there is currently a lack of highly specific clinical diagnostic methods, resulting in frequent clinical misdiagnosis and missed diagnosis.

Anticyclic citrullinated peptide (CCP) antibody is a type of autoantibody mainly present in serum of RA patients [2, 3]. Studies have confirmed that the sensitivity of anti-CCP antibody is basically the same as that of the rheumatoid factor (RF), but its specificity is higher [4]. Therefore, anti-CCP antibody is currently recognized as one of the serological markers with high sensitivity and specificity in the diagnosis of RA.

Antikeratin antibody (AKA) was an RA-specific antibody discovered in RA serum by Young et al. [5]. AKA has high specificity but poor sensitivity in the prediction of RA. Previous studies have found that the specificity of AKA in the diagnosis of RA is as high as 79–100%, while the sensitivity is 20–80% [6–8]. A meta-analysis of 2350 RA patients and 2067 control subjects showed that AKA had a sensitivity of 0.46 (95% CI 0.44–0.48) and a specificity of 0.94 (95% CI 0.93–0.95) for the diagnosis of RA, the diagnostic odds ratio was 15.86 (95% CI 9.48–26.52), and the area under the curve (AUC) was 0.7194 [9]. APF and AKA antibodies target the same antigen, epithelium filaggrin [10]. This antigen is also commonly used in the diagnosis of RA. A study showed that the sensitivity of APF antibody detection in predicting RA was 66.67%, and the specificity was also as high as 81.40% [6].

In this study, we collected the clinical data of 249 RA patients and 149 control groups in Yunnan province; by analyzing and studying the risk factors of RA in Yunnan, we hope to provide reference for the prevention of RA in Yunnan. In addition, a number of studies have shown that RA is an independent risk factor for cardiovascular disease [11], and studying RA risk factors can indirectly prevent the occurrence of cardiovascular disease and reduce the risk of the population.

## 2. Subjects and Methods

### 2.1. Clinical Information

A total of 249 RA patients admitted to the First People's Hospital of Yunnan Province from January 2014 to February 2022 were selected. Inclusion criteria were as follows: age 18 and above; the diagnosis of RA refers to the diagnostic criteria revised by the American College of Rheumatology (ACR) in 1987; and the clinical medical records were kept intact. Exclusion criteria were as follows: patients with Sjögren's syndrome, systemic lupus erythematosus, or osteoarthritis; patients in the acute infection phase; transaminase increased more than 3 times; glomerular filtration rate <15 ml/min*∗*1.73 m^2^; and malignant tumor patients, patients with hematopoietic system diseases or endocrine system disease patients. Another 149 healthy subjects were selected as the control group. Patients with RA were excluded, and they were all over 18 years old, and clinical information was complete.

### 2.2. Collection of Clinical Information

The clinical information we collected in this study included the subjects' age, sex, history of diabetes mellitus, and history of hypertension. Clinical data were derived from patients' diagnosis and treatment data or electronic medical records. The test results of serum anti-CCP antibody, AKA and APF, were collected from the laboratory database. Anti-CCP ≥ 30.0AU/mL was positive, and anti-CCP<30.0AU/mL was anti-CCP negative. Criteria for AKA positive: the epithelial stratum corneum in the frozen section of rat esophagus (middle 1/3) showed typical lamellar and linear stratified homogeneous fluorescent staining. AKA negative criteria: atypical punctate or flaky stratum corneum, the stratum corneum, and other epithelial layers (lamina propria and mucosal layer) showed diffuse full-thickness fluorescence. Criteria for APF positive: homogeneous round and oval fluorescent particles of different sizes and numbers appeared around the nucleus of human buccal mucosa epithelial cells.

### 2.3. Statistical Analysis

The frequencies (%) were used to represent categorical variables, and the *χ*^2^ test was used to compare the significance of differences between groups. Logistic regression was used to analyze the risk factors of RA after adjusting for other confounding factors. The receiver operating curve (ROC) was used to analyze the efficacy of anti-CCP levels in predicting RA, and the sensitivity and specificity were also calculated. All statistical analysis procedures were performed on the SPSS 26.0 statistical software (SPSS Inc, Chicago, IL). All assays were two-tailed, and *p* < 0.05 indicated a statistically significant difference.

## 3. Results

### 3.1. Univariate Analysis of the RA Risk

The clinical data of 249 RA patients and 149 controls included in this study are given in Table 1. The results showed that there were statistically significant differences in the age, hypertension, and diabetes proportions of RA patients and the control group (*p* < 0.05); however, there was no statistically significant difference in sex between the two groups (*p* > 0.05).

### 3.2. Anti-CCP Levels in RA Patients and Controls

We analyzed serum anti-CCP levels in RA patients and controls, and the results showed that serum anti-CCP levels in RA patients (30.56 (8.77, 390.22) AU/mL) were significantly higher than those in controls (6.58 (3.42, 14.54) AU/mL), and the difference was statistically significant (*p* < 0.01) (Figure 1(a))). The receiver operating curve (ROC) was used to analyze the power of serum anti-CCP in diagnosing RA. The results showed that the AUC of serum anti-CCP level in diagnosis of RA was 0.76 (95% CI: 0.72–0.81, *p* < 0.01), the sensitivity was 85.23%, the specificity was 61.45%, and the cutoff value was 18.07 AU/mL (Figure 1(b))).

### 3.3. Detection Results of Anti-CCP, AKA, and APF

The comparison of anti-CCP positive rates, AKA positive rates, and APF positive rates between RA patients and the controls is given in Table 2. The analysis results showed that the positive rate of AKA in RA patients was 33.73%, which was significantly higher than the controls (4.03%), and the difference was statistically significant (*p* < 0.001). The positive rate of APF in RA patients was 43.37%, which was also significantly higher than that in the controls (6.04%), and the difference was statistically significant (*p* < 0.001).

### 3.4. Multivariate Logistic Regression Analysis

Logistic regression was used to analyze the risk factors of RA, and after adjusting for confounding factors, we found that anti-CCP positive, AKA positive, and APF positive were all independent risk factors for RA (OR = 20.24, 95% CI: 9.36–43.77, *p* < 0.01; OR = 4.33, 95% CI: 1.62–11.60, *p* < 0.01; and OR = 5.28, 95% CI: 2.33–11.99, *p* < 0.01) (Table 3).

## 4. Discussion

Rheumatoid arthritis (RA) is an autoimmune disease with significant clinical heterogeneity [12]. There are various treatments for RA, including antirheumatic drugs, glucocorticoids, NSAIDs, and inflammatory cytokine inhibitors, and their treatment regimens are often associated with different clinical effects and characteristics [13, 14]. Due to the pathophysiological heterogeneity of RA, RA patients have a certain individualized response to standard treatment, resulting in poor prognosis [15]. Disease progression leads to loss of patient function, reduced quality of life, and increased morbidity and mortality in the overall population [16]. More importantly, RA also affects organs other than joints, such as the lungs, skin, and cardiovascular system [17, 18]. Therefore, exploring early intervention measures for RA may be of great significance for improving the disease status of RA patients.

Early and accurate diagnosis and treatment of RA can improve disease prognosis. Anti-CCP antibodies highly specific for RA are derived from inflamed synovium [19]. A recent study of 37 RA patients and 91 non-RA controls found that the serum anti-CCP antibody level in RA patients was significantly higher than those in the controls, the sensitivity of serum anti-CCP antibody in predicting RA was 83.7%, and the specificity was as high as 95.6% [20]. This indicates that the serum anti-CCP antibody level is a valuable potential diagnostic indicator of RA. Another study on 191 RA patients and 132 controls showed that the sensitivity of anti-CCP antibody positive diagnosis of RA was 47.1%, and the specificity was 97.4%; this proved that the sensitivity of anti-CCP antibody in diagnosing RA was not high, but the specificity is fully expected.

Our results showed that anti-CCP positivity was an independent risk factors for RA after adjusting for confounding factors, indicating that serum anti-CCP antibodies may be associated with the occurrence of RA. The AUC of the serum anti-CCP level in the diagnosis of RA was 0.76, the sensitivity was 85.23%, and the specificity was 61.45%. We know that the emergence of anti-CCP antibodies is earlier than the onset of RA, which is the early process of RA development [21, 22]. In recent years, anti-CCP antibody has been used as a marker molecule for RA [23]. Since the development of the enzyme-linked immunosorbent assay (ELISA) kit for anti-CCP antibody, researchers are increasingly concerned about the role of this antibody in the diagnosis and prognosis of RA [24, 25]. It has basically become a consensus that anti-CCP has low sensitivity and high specificity in diagnosing RA. The underlying reasons may be that such autoantibodies are pathogenic before symptoms appear or they may be incidental phenomena caused by subclinical synovial inflammation. However, despite these difficulties, these antibodies may be useful predictive markers in very early stage disease.

In addition, we found that the positive rates of AKA and APF were as high as 33.73% and 43.37% in RA patients, while only 4.03% and 6.04% in the controls. After adjusting for confounding factors, it was found that AKA positive and APF positive were independent risk factors for the occurrence of RA. It suggested that AKA and APF were potentially valuable indicators in RA risk assessment. In this study, we analyzed risk factors for the development of RA, although we included RA patients and controls with differences in age, proportion of hypertensive patients, and diabetic patients; after adjusting for these confounding factors, we found that the risk of developing RA was also significantly increased when accompanied by hypertension or diabetes mellitus, indicating that cardiovascular diseases such as hypertension, diabetes, and metabolic abnormalities were risk factors for RA.

This study also has some shortcomings. First, the lack of quantitative detection data of AKA and APF limits our use of AKA and APF as a diagnosis of RA. Second, data on traditional risk factors such as family history, smoking, alcohol consumption, and hyperlipidemia are lacking. Third, further research is needed on the related mechanism of anti-CCP antibodies, AKA and APF, and the development of RA. In addition, in this study, we did not further analyze the sensitivity and specificity of AKA and APF in the diagnosis of RA and did not analyze the value of combined diagnosis, which is also the inadequacy of our study. Based on the data of anti-CCP, AKA, and APF, we estimated that the minimum sample sizes required for RA patients and controls in this study were 13 cases, 8 cases, 25 cases, 15 cases, 18 cases, and 11 cases, respectively [26]. Finally, this study needs to be validated in a large sample size.

## 5. Conclusion

In conclusion, our study demonstrated that anti-CCP positivity, AKA positivity, and APF positivity were independent risk factors for the development of RA. The serum anti-CCP level has high sensitivity but low specificity in diagnosis of RA. The value of combined anti-CCP antibody, AKA and APF, in the diagnosis of RA needs to be further studied.

## Figures and Tables

**Figure 1:** Analysis of serum anti-CCP levels. (a) Comparison of serum anti-CCP levels between RA patients and controls. (b) Receiver operating curve (ROC) of serum anti-CCP levels in predicting RA.

**Table 1:** The results of univariate analysis of RA risk (*n* (%)).

Index	RA patients (*n* = 249)	Controls (*n* = 149)	*χ* ^2^ value	*P* value
Age (years)				
<60	173 (69.48)	122 (81.88)	7.474	0.006
≥60	76 (30.52)	27 (18.12)		

Sex				
Male	73 (29.32)	43 (28.86)	0.009	0.922
Female	176 (70.68)	106 (71.14)		

Hypertension				
Yes	56 (22.49)	10 (6.71)	16.777	<0.001
No	193 (77.51)	139 (93.29)		

Diabetes mellitus				
Yes	42 (16.87)	9 (6.04)	9.781	0.002
No	207 (83.13)	140 (93.96)		

RA, rheumatoid arthritis.

**Table 2:** Comparison of positive rates of AKA and APF between the RA patients and controls (*n* (%)).

	RA patients (*n* = 249)	Controls (*n* = 149)	*χ* ^2^ value	*P* value
Anti-CCP				
Positive	125 (50.20)	8 (5.37)	84.206	<0.001
Negative	124 (49.80)	141 (94.63)		

AKA				
Positive	84 (33.73%)	6 (4.03%)	47.014	<0.001
Negative	165 (66.27%)	143 (95.97%)		

APF				
Positive	108 (43.37%)	9 (6.04%)	62.599	<0.001
Negative	141 (56.63%)	140 (93.96%)		

RA, rheumatoid arthritis; CCP, cyclic citrullinated peptide; AKA, antikeratin antibody; APF, antiperinuclear factor.

**Table 3:** Logistic regression analysis of risk factors for RA.

Factors	B	Standard error	Wald	*P* value	OR (95% CI)
Male	0.32	0.28	1.34	0.25	1.38 (0.80–2.39)
Age ≥ 60	0.44	0.31	2.07	0.15	1.56 (0.85–2.85)
Hypertension	1.56	0.39	16.17	<0.01	4.76 (2.23–10.18)
Diabetes mellitus	1.01	0.44	5.23	0.02	2.75 (1.16–6.52)
Anti-CCP positive	3.01	0.39	58.44	<0.01	20.24 (9.36–43.77)
AKA positive	1.47	0.50	8.48	<0.01	4.33 (1.62–11.60)
APF positive	1.67	0.42	15.87	<0.01	5.28 (2.33–11.99)

CCP, cyclic citrullinated peptide; AKA, antikeratin antibody; APF, antiperinuclear factor; OR, odds ratio; CI, confidence interval.

## Data Availability

The data used to support the findings of this study are available from the corresponding author upon request.
